This article has been retracted.

# Knowledge, attitude, and practice towards enhanced recovery after surgery among patients underwent thoracoscopy surgery

**DOI:** 10.1371/journal.pone.0309821

**Published:** 2024-09-04

**Authors:** Yinping Huang, Xingbang Wang, Jiajia Li, Qing He, Rui Wang

**Affiliations:** Lu’ an People’ s Hospital General thoracic surgery, Lu’ an, China; Ministry of Health, General Health Directorate of Raparin and University of Raparin, IRAQ

## Abstract

**Objective:**

Thoracoscopy has gained extensive utilization in managing pleural disorders, and enhanced recovery after surgery (ERAS) can improve patients’ prognosis and expedite post-surgical recovery. This study aimed to investigate the knowledge, attitudes, and practices (KAP) towards ERAS among patients underwent thoracoscopy surgery.

**Methods:**

This cross-sectional study was conducted between September 2022 and August 2023, among patients underwent thoracoscopy surgery in 6 Secondary or Tertiary hospitals in the author’s area. Demographic characteristics and KAP scores were collected by questionnaires, and clinical data were extracted from medical records.

**Results:**

A total of 309 valid questionnaires were collected, with 165 (53.40%) males and 202 (65.37%) aged ≤65 years old. The mean scores for KAP were 28.92±7.21 (possible range: 9–45), 53.60±6.73 (possible range: 13–65), and 43.45±5.50 (possible range: 10–50), respectively. SEM confirmed the positive associations between knowledge and attitude (β = 0.108, P = 0.019), knowledge and practice (β = 0.096, P = 0.004), and attitude and practice (β = 0.438, P<0.001). However, the KAP were found not associated with prognosis.

**Conclusion:**

Patients underwent thoracoscopy surgery showed moderate knowledge, positive attitude, and appropriate practice towards ERAS. Preoperative education, personalized counseling, peer support groups, peer support groups, and follow-up care were recommended in further clinical practice.

## Introduction

Thoracoscopy, a minimally invasive surgical approach facilitating visualization and treatment within the pleural cavity, has garnered significant prominence in modern healthcare [1]. This technique has revolutionized diagnostic and therapeutic approaches for various thoracic conditions [2]. Through the utilization of thoracoscope introduced via minor incisions, this method offers reduced invasiveness, shorter hospitalization, and faster recovery compared to traditional open surgeries [3]. Globally, the escalating adoption of thoracoscopy is attributed to its effectiveness and patient-centric benefits [4]. Notably in China, thoracoscopy has been widely used for addressing pleural diseases, including tuberculous pleural effusion, malignant pleural effusion, and spontaneous pneumothorax [5]. This trend accentuates the need to explore factors impacting patients’ experiences and outcomes after undergoing thoracoscopy. Nonetheless, beyond its surgical advantages, thoracoscopy can also lead to postoperative discomfort, physical limitations during recovery, and psychological stress due to surgery-related anxiety [6]. Therefore, these complications can detrimentally affect patients’ quality of life and mental well-being, which highlighted the importance of appropriate support and management strategies.

Enhanced Recovery after Surgery (ERAS) represents a comprehensive approach aimed at optimizing patient outcomes and expediting post-surgery recovery [7]. This multifaceted strategy spans preoperative preparation to postoperative care, and is collectively designed to mitigate stress responses, promote rapid functional recovery, and reduce complications. Currently, the integration of ERAS protocols has demonstrated remarkable success across surgical specialties, including thoracoscopy [8]. Tailoring ERAS for thoracoscopy holds potential for shorter hospital stays, fewer complications, and heightened patient satisfaction. Furthermore, knowledge of ERAS among patients, coupled with their attitudes toward thoracoscopy implementation, can substantially influence its adoption. Therefore, the knowledge, attitudes, and practices (KAP) study serves as a suitable methodology to explore the acceptance of ERAS and determine areas of interventions. However, KAP studies of ERAS have mainly focused on medical personnel. For instance, a Chinese study revealed knowledge deficiency among pediatric surgical nurses regarding postoperative recovery and preoperative preparation [9]. Additionally, health professionals exhibited positive attitude toward ERAS but acknowledged its complexity and challenges [10]. However, the dearth of KAP study of ERAS among patients undergoing thoracoscopy still exists in China.

Therefore, this study aimed to explore the KAP towards ERAS among patients underwent thoracoscopy surgery. It was hypothesized that: 1) participants’ knowledge could positively influence their attitudes; 2) participants’ knowledge could positively influence their ERAS practice; and 3) participants’ attitudes could positively influence ERAS practice.

## Methods

### Study design and participants

This cross-sectional study was conducted between September 2022 and August 2023, among patients underwent thoracoscopy surgery in 6 Secondary or Tertiary hospitals in the author’s area. Patients who underwent thoracoscopy surgery and received perioperative nursing on the concept of ERAS were included. Inclusion criteria included: 1) Inpatients scheduled for thoracoscopy surgery; 2) Willingness to participate and signed informed consent; 3) Age ≥ 18 years. Exclusion criteria included: 1) Patients discontinuing surgery for various reasons; 2) Patients necessitating open surgery due to medical conditions; 3) Patients with severe liver, kidney, or hematological diseases; 4) Patients with concurrent psychiatric disorders; 5) Patients directly transferred to ICU postoperatively. Ethical approval was granted by the Medical Ethics Committee of the author’s Hospital, and all participants provided informed consent.

### Questionnaire

The questionnaire was designed based on previous studies [11–14]. And revisions were made based on feedback from five senior experts, the similar or repeated questions were deleted and questions that were not clearly formulated were refined to guarantee content validity. And a pilot study among 50 participants was conducted, with Cronbach’s α coefficient of 0.9359, indicate a good internal consistency.

The final questionnaire was in Chinese, and comprised four dimensions: demographic characteristics, knowledge, attitude, and practice (supplementary materials). The demographic characteristics included 11 items, including age, gender, residence, education, occupation, monthly income, marital status, smoking, alcohol consumption, underlying medical conditions, and medical insurance. The knowledge, attitude, and practice dimensions employed a five-point Likert scale. In the knowledge dimension, 9 questions were posed, with 5 points assigned to "Very familiar", 4 points to "Familiar", 3 points to "Recognizable", 2 points to "Unfamiliar", and 1 point to "Very unfamiliar". The total score of the knowledge dimension ranged from 9 to 45 points. The attitude dimension encompassed 13 questions, with 5 points indicating "Strongly agree", 4 points for "Agree", 3 points for "Neutral", 2 points for "Disagree", and 1 point for "Strongly disagree". The total score of attitude dimension ranged from 13 to 65 points. The practice dimension consisted of 11 questions, with the 6^th^ question analyzed descriptively only. For the remaining 10 questions, 5 points corresponded to "Always", 4 points to "Frequently", 3 points to "Sometimes", 2 points to "Occasionally", and 1 point to "Never". The total score of the practice dimension ranged from 10 to 50 points. The overall KAP scores were categorized according to modified Bloom’s cutoff: respondents scoring between 80–100% were deemed to possess good knowledge, positive attitude, and appropriate practice; 60–79% as moderate; and less than 60% as poor knowledge, negative attitude, and inappropriate practice [15].

### Data collection

The electronic questionnaire was generated by the *“Sojump” platform (www.wjx.cn)*, and were distributed via QR codes. The questionnaires were disseminated to patients when they had received ERAS education before thoracoscopy surgery. In instances where elderly patients lacked smartphones, access to paper-based surveys or assistance from family members using smartphones was facilitated. During the survey, research aides were present to aid participants grappling with comprehension. For individuals encountering difficulties with responses, staff members facilitated question presentation and response recording.

The clinical characteristics were also collected, including patients’ surgery type, surgery durations, intraoperative blood loss, ASA. Surgery type was categorized into pulmonary lobectomy and others (including fracture fixation, exploratory thoracotomy, and drainage). And the prognosis data were also collected, including postoperative bed rest time, hospital stay, and complications (including pneumonia, lung collapse, anastomotic leakage, wound infection, and wound dehiscence).

### Statistical analysis

Statistical analysis was conducted by SPSS 26.0 (IBM, Armonk, NY, USA) and AMOS 23.0 (IBM, Armonk, NY, USA) software. Continuous variables were presented as means ± standard deviation (SD), and compared by ANOVA or Student’s t test. And the categorical variables were expressed as n (%). Pearson’s correlation analysis and structural equation modeling (SEM) were conducted to explore correlation among KAP. Univariate and multivariate logistic and linear regressions were conducted to explore the association between KAP and prognosis. Statistical significance was considered as a two-sided P <0.05.

## Results

A total of 389 questionnaires were gathered. Following exclusions of 37 questionnaires due to insufficient response time, 32 due to incomplete data, and 11 due to logical inconsistencies, 309 valid questionnaires was retained. The majority of participants were male (53.40%), ≤65 years old (65.37%), rural residents (64.40%), educated up to middle school (74.76%), married (92.23%), categorized as ASA classification II (81.88%), and received pulmonary lobectomy (76.05%). Additionally, 39.48% were civil servants, and 41.10% had a monthly income <2,000 yuan **(Table 1)**.

**Table 1:** Demographic characteristics of participants and KAP score distribution.

Characteristics	N (%)	Knowledge (mean ± SD)	*P*	Attitude (mean ± SD)	*P*	Practice (mean ± SD)	*P*
**Total**		28.92±7.21		53.60±6.73		43.45±5.50	
**Gender**			0.911		0.252		0.201
Male	165 (53.40)	28.87±7.41		54.01±6.44		43.82±5.07	
Female	144 (46.60)	28.97±7.01		53.13±7.04		43.02±5.93	
**Age, years**			0.140		0.968		0.399
≤65	202 (65.37)	29.36±7.21		53.58±±7.05		43.26±5.86	
>65	107 (34.63)	28.08±7.18		53.62±6.10		43.81±4.74	
**Residence**			<0.001		0.785		0.940
Rural	199 (64.40)	27.71±7.43		53.52±6.94		43.47±5.54	
Urban or suburban	110 (35.60)	31.09±6.27		53.74±6.35		43.42±5.45	
**Education**			<0.001		0.823		0.183
Middle school or below	231 (74.76)	27.74±7.27		53.55±6.90		43.21±5.61	
High school or above	78 (25.24)	32.38±5.83		53.74±6.22		44.17±5.13	
**Occupation**			<0.001		0.864		0.188
Production worker	77 (24.92)	31.40±6.17		53.86±6.59		44.43±5.07	
Civil servant	122 (39.48)	29.26±6.57		53.35±6.74		43.23±5.75	
Others	110 (35.60)	26.79±7.96		53.68±6.86		43.01±5.46	
**Marital status**			0.618		0.698		0.666
Married	285 (92.23)	28.21±6.53		53.08±6.06		43.92±5.60	
Unmarried/divorced/widowed	24 (7.77)	28.98±7.28		53.64±6.79		43.41±5.50	
**Monthly income, yuan**			0.015		0.238		0.136
<2,000	127 (41.10)	28.08±6.71		52.68±6.39		43.24±5.55	
2,000–5,000	120 (38.83)	28.47±7.83		54.28±6.80		42.96±5.37	
5,000–10,000	42 (13.59)	31.76±6.32		54.40±6.69		44.52±5.45	
>10,000	20 (6.48)	30.95±6.79		53.60±8.22		45.50±5.63	
**Smoking**			0.351		0.625		0.354
Yes	36 (11.65)	27.86±7.47		54.11±6.91		43.43±5.52	
No	273 (88.35)	29.05±7.18		53.53±6.71		44.25±5.32	
**Alcohol consumption**			0.036		0.282		0.568
Yes	69 (22.33)	30.52±6.09		52.83±6.49		43.12±5.28	
No	240 (77.67)	28.45±7.45		53.82±6.79		43.55±5.56	
**Underlying medical conditions**			0.045		0.874		0.520
Yes	140 (45.31)	28.01±7.55		53.53±6.57		43.23±5.17	
No	169 (54.69)	29.66±6.86		53.65±6.88		43.63±5.76	
**Medical insurance type**			0.162		0.004		0.121
Yes	303 (98.06)	29.00±7.22		53.75±6.61		43.52±5.44	
No	6 (1.94)	24.83±6.18		45.83±8.91		40.00±7.72	
**ASA classification**			0.301		0.270		0.364
I	22 (7.12)	31.27±6.85		52.68±8.19		43.36±5.09	
II	253 (81.88)	28.65±7.27		53.66±6.69		43.62±5.35	
III	32 (10.35)	29.25±7.03		53.44±5.94		42.16±6.73	
IV	2 (0.65)	31.50±4.95		58.50±9.19		43.50±9.19	
**Surgery**			0.850		0.626		0.659
Pulmonary lobectomy	235 (76.05)	28.93±7.35		53.48±6.81		43.49±5.64	
Others	74 (23.95)	28.88±6.80		53.97±6.5		43.34±5.07	

*: including fracture fixation, exploratory thoracotomy, and drainage

The participants had an average knowledge score of 28.92±7.21 (possible range: 9–45). Urban and suburban residents (P<0.001), individuals with a high school education or above (P<0.001), those engaged as production workers (P<0.001), participants with monthly income ranging between 5,000–10,000 yuan (P = 0.015), individuals who consumed alcohol (P = 0.036), and those without underlying diseases (P = 0.045) were likely to achieve higher knowledge scores **(Table 1)**. In the knowledge section, the rates of "Very familiar" and "Familiar" ranged from 29.45% to 52.10%. Specifically, 52.10% possessed knowledge about the early postoperative activity requirements within ERAS **(K6)**. In contrast, a mere 29.45% of participants were acquainted with ERAS, encompassing its definition and primary research content **(K1)**. Additionally, only 30.74% of participants were informed about the requisites for implementing ERAS **(K3) (S1 Table)**.

The participants had an attitude score of 53.60±6.73 (possible range: 13–65). Participants with medical insurance displayed significantly higher attitude scores (P = 0.004) **(Table 1)**. In the attitudes section, the rate of positive responses varied between 66.34% and 90.30%. A substantial proportion (90.30%) of participants showcased a positive attitude towards prioritizing the timely seeking of healthcare experts’ assistance in case of postoperative incisional pain, instead of enduring the discomfort **(A10)**. Conversely, the smallest proportion of participants (66.34%) concurred with the sentiment that surgical procedures trigger emotional anxiety within them **(A1)**. Similarly, a mere 73.14% agreed that unless it affects the surgical procedure, minimizing the fasting duration before the operation takes precedence **(A4) (S2 Table)**.

The participants displayed a mean practice score of 43.45±5.50 (possible range: 10–50) **(Table 1)**. There was variability in practice adherence among participants, with rates ranging from 89.32% to 94.17%. The highest proportion (94.17%) of participants adhered to prescribed fasting and abstention from drinking before surgery under medical guidance **(A4)**, as well as collaborated with healthcare professionals to discontinue smoking and alcohol intake prior to the procedure when applicable **(A6)**. In contrast, the lowest proportion of participants (89.32%) engaged with medical personnel for participation in preoperative respiratory exercises **(A3)**. Similarly, 89.32% of participants endorsed the use of relaxation techniques and prompt nursing assistance in case of postoperative incisional pain **(A10) (S3 Table)**.

Pearson’s correlation analysis revealed significantly positive correlations among knowledge and attitude (r = 0.127, P = 0.026), as well as knowledge and practice (r = 0.222, P<0.001). Furthermore, attitude was positively correlated with practice (r = 0.489, P<0.001) **(Table 2)**. The SEM results confirmed that knowledge was positively associated with attitude (β = 0.108, P = 0.019) and practice (β = 0.096, P = 0.004). Moreover, attitude was positively associated with practice (β = 0.438, P<0.001), which was consistent with the main findings from Pearson correlation analysis **(Table 3, Fig 1)**.

**Fig 1:** Structural equation model showing the associations between demographic characteristics and KAP. All variables are observed variables. Direction of causality is indicated by single-headed arrows. The standardized path coefficients are presented alongside the arrows.

**Table 2:** Pearson correlation analysis of KAP scores among participants.

	Knowledge	Attitude	Practice
Knowledge	1		
Attitude	0.127 (P = 0.026)	1	
Practice	0.222 (P<0.001)	0.489 (P<0.001)	1

**Table 3:** The estimates of SEM.

Model paths	Estimate	Standard error	*P*
Knowledge → Attitude	0.108	0.046	0.019
Attitude → Practice	0.438	0.053	<0.001
Knowledge → Practice	0.096	0.034	0.004

The mean intraoperative blood loss was 96.22±8.13 ml, the mean postoperative bed rest time was 25.47±0.89 hours, the mean postoperative hospital stay was 9.15±0.33, and 105 (33.98%) patients experienced postoperative complications. And the most frequently complication was lung infection (52 [16.83%]), followed by the hypoproteinemia (36 [11.65%]), and pneumothorax (25 [8.09%]) **(S4 Table)**. However, the multivariate logistic and linear regression revealed that the KAP were not associated with postoperative bed rest time, hospital stay, or complications after adjusted for factors including alcohol consumption, ASA classification, surgery duration, and surgery types **(S5–S7 Tables)**.

## Discussion

The study demonstrated that patients undergoing thoracoscopy displayed moderate knowledge, positive attitudes, and appropriate practice to ERAS. Moreover, positive associations were identified among KAP scores. These findings might offer valuable insights for designing healthcare interventions and educational campaigns for enhancing ERAS-related KAP.

This study firstly explored the KAP towards ERAS among patients underwent thoracoscopy surgery. The previous KAP studies towards ERAS mainly focus on the medical professionists. Specifically, a study from China demonstrated knowledge gaps in preoperative preparation and postoperative recovery among surgical nurses [9]. Similarly, another research in Pakistan revealed that the majority of surgical residents struggled to identify and implement ERAS protocol [16]. In contrast, patients underwent thoracoscopy surgery exhibited heightened KAP levels in our study. This improvement might stem from heightened awareness, better training, and enhanced healthcare provider-patient communication, as well as heterogeneity in study design and questionnaire items. The findings potentially underscored the positive influence of healthcare education strategies, which could contribute to a more informed patient population regarding ERAS practices.

In the knowledge dimension, 52.10% of participants was knowledgeable about the early postoperative requirements of ERAS. This finding indicated a relatively robust understanding of the importance of postoperative activities among patients underwent thoracoscopy surgery. In contrast, only 29.45% of participants were acquainted with the overall definition and primary research content of ERAS. This lack of awareness might stem from inadequate dissemination of enhanced recovery in the preoperative and postoperative settings [17]. Given that ERAS involves a holistic strategy encompassing preoperative, intraoperative, and postoperative phases, such a disparity in knowledge underscored the need for targeted educational initiatives to elucidate the core principles and objectives of ERAS [14]. Furthermore, the acknowledgment of requisites necessary for the effective implementation of ERAS was evident in only 30.74% of participants. This lack of awareness could potentially hinder the effective implementation of ERAS protocols, leading to suboptimal surgical outcomes and prolonged recovery periods. Targeted patient education should be developed to provide training on ERAS protocols and address related misunderstandings through doctor-patient communications.

The majority of participants (90.30%) demonstrated positive attitude towards promptly seeking the guidance of healthcare professionals when confronted with postoperative incisional pain, rather than enduring the discomfort. This finding aligned with the principles of patient-centered care, and emphasized the importance of addressing postoperative pain in a proactive and efficient manner [18]. The positive attitude held the potential to contribute to improved patient outcomes and enhanced overall satisfaction with the surgical process. Conversely, the smallest proportion of participants (66.34%) expressed concurrence with the notion that surgical procedures evoke emotional anxiety within them. While surgical anxiety is a common sentiment, the comparatively lower agreement rate suggested that a significant portion of participants either had effective coping mechanisms or viewed the surgical process from a more objective standpoint [19]. This insight prompted further exploration into preoperative psychological preparation, and supported strategies to alleviate anxiety for patients undergoing thoracoscopy. Besides, a modest proportion (73.14%) of participants acknowledged the significance of minimizing fasting periods unless it directly impacted the surgical procedure. Since ERAS emphasized the importance of preoperative nutrition to facilitate postoperative recovery, educational efforts towards rationale behind fasting guidelines and their implications for surgical outcomes were necessary [20].

The highest proportion (94.17%) of participants adhered to prescribed fasting and abstention from smoking and alcohol intake in the practice dimension. This underscored participants’ recognition of the detrimental effects of these habits on surgical outcomes. It was worth noting that cessation of smoking and alcohol consumption is vital in mitigating postoperative complications and fostering conducive environment for recovery [21]. Conversely, a comparatively lower adherence rate (89.32%) was observed in participants’ engagement with medical personnel in preoperative respiratory exercises. Given the significance of such exercises in maintaining optimal lung function postoperatively, addressing potential barriers to engagement in these practices could be beneficial [22]. Similarly, the endorsement of relaxation techniques and the prompt seeking of nursing assistance was reported by 89.32% of participants, suggestive of proactive management in postoperative incisional pain.

In contrast to a prior study where patients undergoing thoracoscopic surgery lobectomy were discharged within 4 days [23], patients in our study experienced a longer postoperative hospital stay (9.15±0.33 days). Several factors may contribute to this extended duration. Firstly, a majority of patients underwent pulmonary lobectomy, which is a treatment modality for severe lung diseases. Additionally, the management of potential complications such as lung infection, pneumothorax, and hypoproteinemia could have prolonged hospitalization. However, direct comparisons of hospital stay lengths are challenging due to variations in discharge criteria among studies. The positive associations among KAP scores highlighted the necessity of targeted interventions and educational programs to augment ERAS-related KAP among patients undergoing thoracoscopy. This observation could be ascribed to the influence of knowledge on attitudes and practices of ERAS, in accordance with the theory of planned behavior, where attitudes and practices were shaped by the perception of behavioral consequences [24]. Besides, the lack of significant associations between KAP scores and clinical outcomes was found. One plausible explanation was that the effectiveness of ERAS might not be contingent upon the patients’ KAP. Instead, it might rely more heavily on the implementation of ERAS by healthcare providers, such as optimized anesthesia, minimal incision techniques, and early mobilization. Besides, all patients completed the questionnaire after receiving education about ERAS, which contributed to the elevated KAP scores and thus masked their relationships with clinical outcomes. This underscored the importance of integrating ERAS education into preoperative care for patients undergoing thoracic surgery and similar surgeries. Standardization of ERAS education may also facilitate comparisons across different patient populations, enabling researchers to evaluate the impact of education on patient outcomes more rigorously in future studies.

This study had several limitations. Firstly, its confined scope to a single region with limited sample size restricted the generalizability of the findings. Nonetheless, the findings provided valuable insights into the present KAP status of patients undergoing thoracoscopy towards ERAS. Secondly, the KAP scores could be influenced by social desirability bias, possibly leading to an overestimation of the scores. Participants might tend to provide responses that aligned with social norms rather than accurately reflecting their behaviors and knowledge [25]. Thirdly, the limited items of early postoperative outcomes (postoperative complications, postoperative bed rest time and duration of hospital stay) were collected, which cannot comprehensively grasp the relationships between KAP and early postoperative outcomes. Therefore, the observed findings should be taken with caution. Fourthly, several variables, such as previous surgical procedure, nutritional status and duration of pleural drainage, were not included in the questionnaire. The missing information can impede the investigation into the determinants of clinical outcomes, highlighting the need for future studies involving a larger cohort of phenotyped individuals.

## Conclusions

In conclusion, patients underwent thoracoscopy surgery showed moderate knowledge, positive attitudes, and appropriate practice towards ERAS. Based on the identified gaps in KAP items, we recommend further development of preoperative education, personalized counseling, peer support groups, and follow-up care to enhance the prognosis and quality of life for individuals undergoing thoracoscopy.

## Supporting information

S1 Checklist STROBE statement—checklist of items that should be included in reports of *cross-sectional studies*. (DOC)

S1 Table Distribution of knowledge dimension responses. (DOCX)

S2 Table Distribution of attitude dimension responses. (DOCX)

S3 Table Distribution of practice dimension responses. (DOCX)

S4 Table The patients’ prognosis characteristics. (DOCX)

S5 Table Univariate and multivariate logistic regression analysis of postoperative complications. (DOCX)

S6 Table Univariate and multivariate linear regression analysis of postoperative bed rest time. (DOCX)

S7 Table Univariate and multivariate linear regression analysis of duration of hospital stay. (DOCX)

S1 Data (XLSX)

S1 Questionnaire (DOC)
